The article "Is Generalized Maternal Optimism or Pessimism During Pregnancy Associated with Unplanned Cesarean Section Deliveries in China?" was published in 2011. Journal: J Pregnancy.

# Is Generalized Maternal Optimism or Pessimism During Pregnancy Associated with Unplanned Cesarean Section Deliveries in China?

**DOI:** 10.1155/2010/754938

**Published:** 2011-01-05

**Authors:** Cheryl A. Moyer, Yasmin Elsayed, YuChun Zhu, Yumei Wei, Cyril M. Engmann, Huixia Yang

**Affiliations:** ^1^Global REACH, Medical School, University of Michigan, 5115 Med Sci 1, 1301 Catherine Street, Ann Arbor, MI 48109, USA; ^2^Minority and Health Disparities International Research Training Program (MHIRT), Center for Human Growth and Development, University of Michigan, MI 48109, USA; ^3^Department of Medical Education, Medical School, University of Michigan, MI 48109, USA; ^4^Department of Obstetrics and Gynecology, Peking University First Hospital, 8 Xishiku Street, Xicheng District, Beijing 100034, China; ^5^Division of Neonatal-Perinatal Medicine, Department of Pediatrics, University of North Carolina at Chapel Hill, CB 7596, 4th Floor, UNC Hospitals, Chapel Hill, NC 27599-7596, USA

## Abstract

This research examines whether maternal optimism/pessimism is associated with unplanned Cesarean section deliveries in China. If so, does the association remain after controlling for clinical factors associated with C-sections? A sample of 227 mostly primiparous women in the third trimester of pregnancy was surveyed in a large tertiary care hospital in Beijing, China. Post-delivery data were collected from medical records. In bivariate analysis, both optimism and pessimism were related to unplanned c-section. However, when optimism and pessimism were entered into a regression model together, optimism was no longer statistically significant. Pessimism remained significant, even when adjusting for clinical factors such as previous abortion, previous miscarriage, pregnancy complications, infant gestational age, infant birthweight, labor duration, birth complications, and self-rated difficulty of the pregnancy. This research suggests that maternal mindset during pregnancy has a role in mode of delivery. However, more research is needed to elucidate potential causal pathways and test potential interventions.

## 1. Introduction

Worldwide, Cesarean section rates are increasing [1–3]. Despite recommendations that cesarean section rates not exceed 15% [4, 5], many countries have rates double or even triple that threshold [3]. China—home to one-fifth of the world's population and 12 percent of all births annually [6, 7]—is no different. Data from hospital-based studies in urban China showed c-section rates ranging from 26% to 63% during the late 1990s [8], while a more recent WHO study combining urban and rural populations reported overall c-section rates of 46.2% [3].

Although cesarean section deliveries can be lifesaving for both mothers and their infants when indicated, their overuse is cause for concern due to their association with increased maternal morbidity and mortality, cost, and utilization of sometimes scarce health system resources [3]. Numerous researchers have investigated the predictors of higher than normal cesarean section rates [9–15]. Principal among these include including physician-related factors, insurance-related factors, hospital and health-system factors, and maternal preferences. Additionally, cesarean section rates have also been found to vary by male versus female provider [15], public versus private hospital setting [16–19], adoption and use of clinical guidelines [20], public versus private insurance status [18], and even day of the week and time of day [17, 19, 21] that women present for delivery. Patient race [16], age [22], income [22], and preferences [23] have also been linked to increased c-section rates. 

Although the literature is replete with clinical factors associated with elective and emergency cesarean section, such as advanced maternal age, short maternal stature, heavier infant birthweight, fetal dystress, preeclampsia, prolonged/obstructed labor, or shoulder distocia [8, 24], less is known about psychological factors that affect women who intend to delivery vaginally but ultimately deliver via c-section. It is probable that the vast majority of unplanned cesarean sections are attributable to clinical indications. However, are there potential psychological variables at play as well? And in a country like China, with exceedingly high rates of cesarean section, might the impact of those psychological variables be observable?

This exploratory study was designed to examine the psychological characteristic of dispositional optimism and pessimism in a woman's likelihood of undergoing an unplanned cesarean section delivery in urban China. Dispositional optimism is seen as a relatively stable personality characteristic (a “trait” rather than a “state”) that is associated with general assumptions about positive future outcomes. Dispositional pessimism is the converse: it is a tendency to expect the worst when looking toward future outcomes. A meta-analytic review of the optimism literature from 2009 [25] that examined 83 separate studies found a persistent relationship between optimism and positive health outcomes [25]. In addition, women with higher levels of optimism during pregnancy have been found to have to lower levels of stress, anxiety, and peripartum depression than women with lower levels of optimism [26–29]. Optimism has also been linked to birth outcomes, with one study finding that optimistic women gave birth to larger babies [30], and a second study finding that when gestational age was controlled for, women who were least optimistic during pregnancy when compared to women with higher levels of optimism delivered smaller infants [31]. 

It may seem logical to conclude that if optimism can lead to better health outcomes, pessimism might be detrimental. However, pessimism has been shown to have prophylactic effects in certain circumstances. In particular, pessimism can insulate people from the psychological consequences of failure, including anxiety, depression, and diminished self-esteem [32]. Norem and Cantor [32, 33] found that individuals who expect the worst can sometimes use those expectations to help them better meet the demands of stressful challenges. These “defensive pessimists” engage in active and constructive coping efforts—which may mediate the relationship between pessimism and outcomes [34]. For example, Moyer et al. found that among pregnant women in Ghana, those who were the most pessimistic were more likely to get tested for HIV whereas their optimistic counterparts were less likely to get tested [35]. 

This research aimed to address the following research questions. (1) Is generalized maternal optimism or pessimism (assessed during pregnancy) associated with unplanned cesarean section among women giving birth in a tertiary care hospital in Beijing? (2) If optimism or pessimism is associated with unplanned cesarean section, which is more strongly associated, optimism or pessimism? And (3) if there is a significant relationship between optimism, pessimism, and unplanned cesarean section delivery, is that relationship robust enough to remain significant when clinical factors are included in the model?

## 2. Materials and Methods

### 2.1. Study Site

Data were collected from pregnant women presenting for prenatal care at the obstetric outpatient clinic at the Peking University First Hospital between May and July 2006. As one of the largest and most well-known academic medical centers in Beijing, Peking University First Hospital draws both public and private patients from in and around Beijing. Clinics see an average of 600 pregnant women per week and 3000–3500 deliveries per year.

### 2.2. Patient Population and Data Collection

All research protocols and survey instruments were reviewed and approved by the institutional review boards at the University of Michigan and Peking University. 

Pregnant women in their last trimester of pregnancy who were 18 years old or older attending antenatal care clinic were eligible. Women facing an imminent health crisis, those in active labor, or those being admitted to the hospital were excluded (despite the generally stable nature of optimism and pessimism, those women in active labor were excluded because of concerns about disproportionate reporting of a pessimistic attitude if it was assessed during painful, active labor when compared to assessments obtained during a routine prenatal visit). After describing the study and obtaining verbal approval to continue, research assistants talked patients through an informed consent form, answering any questions the women may have had. All participants signed a written informed consent document and were given a copy to keep. Women were then given a self-administered survey to complete before their appointment. Translators were used when necessary. Surveys were designed to be self-administered, but women were given the option to have the survey administered verbally. 

Data were gathered using paper and pencil forms. Hospital registration numbers were collected from participants to allow for postdelivery followup. Hospital registration numbers were removed from the original survey and replaced with a unique ID number once the registration number was recorded in a separate location for follow-up purposes. Responses from the hard copies of the self-administered surveys were entered into an Excel spreadsheet and cleaned.

### 2.3. Instruments

The survey included administering a demographic and health questionnaire and the Life Orientation Test (LOT-R). 

The *Demographic and Health Questionnaire measured* patient characteristics including age, number of pregnancies, other medical conditions, and self-perceived health status. Women were asked to enumerate any pregnancy complications or symptoms they had during pregnancy, including such things as vaginal bleeding, headaches, swollen hands, troubled vision, preeclampsia, dizzy spells, swollen face, abdominal/belly pain, eclampsia, or other problems. For the purposes of this analysis, these were combined into a single dichotomous variable, and termed maternal complications. Women were also asked to rate their perception of the difficulty of their pregnancy on a scale of 1 to 4, with 1 being “extremely easy” and 4 being “extremely difficult.”

The *Life Orientation Test* (LOT), developed by Sheier and Carver in 1985 [36] and revised in 1994 [37] (*Life Orientation Test—Revised*, or LOT-R), was used to assess dispositional optimism. The LOT-R is one of the most commonly used measures of optimism/pessimism. It uses generalized outcome expectancies to measure dispositional optimism. The LOT-R has been widely validated [38] and used in China [39–46]. It includes 6 scored items and 4 fillers that generate an overall score, as well as two possible subscales: an optimism subscale and a pessimism subscale. The items that make up the optimism subscale are (1) in uncertain times, I usually expect the best; (2) I'm always optimistic about my future and (3) overall, I expect more good things to happen to me than bad. The items that make up the pessimism subscale are (1) if something can go wrong for me, it will; (2) I hardly ever expect things to go the way I would like them to go; (3) I rarely count on good things happening to me. The participant answers each item based on a 5-point scale, with response options ranging from strongly disagree to strongly agree. The pessimism items are reverse scored and then added to the optimism items to create the overall score whereas the subscales are created by summing the items for pessimism and the items for optimism separately. For these analyses, the optimism and pessimism subscales were used separately.

The instrument was pilot tested, and minor modifications were made to ensure comprehension. The survey was translated into Mandarin and back-translated into English by native bilingual speakers. The original and back-translated versions were compared for consistency, and any inconsistencies were resolved by discussion and consensus among the research team.

**Chart Review**

was used to collect data after women had delivered their babies. Mode of delivery was determined, which indicated vaginal delivery with and without forceps, vaginal delivery with and without vacuum extraction, planned cesarean section, or unplanned cesarean section. For the purposes of this analysis, a single dichotomous variable was created to reflect unplanned cesarean section yes/no. Thus women who delivered vaginally or via planned cesarean section were treated as one group, and women undergoing an unplanned or emergency cesarean section were treated as a separate group. Additional data collected from the medical record included gestational age of the infant at delivery, birthweight, labor duration, use of pain medication, 1-minute and 5-minute Apgar scores, and any of a number of delivery or birth complications, including such things as hemorrhage, preeclampsia, intrauterine infection, breech presentation, or delayed labor. For the purposes of this analysis, all of those factors were combined into a single dichotomous variable termed birth complications.

### 2.4. Data Analysis

Chart review Data were entered into a spreadsheet and cleaned. All data were analyzed using SPSS statistical software, Version 17.1 (SPSS Inc, Chicago, IL). Frequencies and basic descriptive statistics were calculated for all variables. Women with complete baseline and chart data (and could thus be included in the larger regression analysis) were compared against those women with incomplete baseline or chart data using Student's *t*-test for continuous variables and Chi Square analysis for categorical variables.

To address Research Question 1, (*is optimism or pessimism associated with unplanned cesarean section delivery?*), bivariate statistics were calculated to determine if optimism or pessimism were independently associated with unplanned cesarean section. Additional demographic and clinical variables were examined to determine if there were factors aside from optimism and pessimism and expected clinical correlates that might be associated with unplanned cesarean section in this population. Bivariate analysis included Student's *t*-tests, ANOVAs, and Chi-Square analyses. 

To address Research Question 2, (*which is more strongly associated with unplanned cesarean section delivery, optimism or pessimism?*) Binary logistic regression analysis was conducted with both optimism and pessimism regressed on unplanned cesarean section (yes/no). Area under the curve analysis was conducted to judge the strength of the model.

To address Research Question 3, *(if there is a significant relationship between optimism, pessimism, and unplanned cesarean section delivery, is that relationship robust enough to remain significant when clinical factors are included in the model?*), binary logistic regression analysis was conducted with optimism and pessimism regressed on unplanned cesarean section (yes/no) with the additional clinical factors of labor duration, birth complications, previous abortion, previous miscarriage, pregnancy complications, gestational age, infant birth weight, and self-rated difficulty of the pregnancy added into the model. Area under the curve analysis was conducted to judge the strength of the model. 

For all analyses a *P* value of  .05 was taken as statistically significant.

## 3. Results

Two hundred fifty-one women were asked to participate, and 227 met our eligibility criteria and agreed to participate (90.4% response rate). Of the 227, 86 had missing items on their surveys or their birth outcomes data were not available in the hospital medical records system.  Table 1 illustrates our sample demographics, comparing the 141 women who were ultimately included in our analysis with the 86 who were excluded. Overall, our sample is one of well-educated Han women in their last trimester of pregnancy who are married and working outside the home. They do not differ significantly from the 86 women excluded from the analysis on any variable aside from education, with excluded women more likely to have lower levels of education (*P*  =  .012). 

Table 2 illustrates the health-related variables reported at enrollment. Again, there were no significant differences found between women included in our analysis and those excluded due to missing data. More than half of our sample has had at least one previous pregnancy that was either spontaneously or electively terminated, and only 2.8 percent of women report having anything other than mild complications in this current pregnancy. The vast majority of women in this study were primiparous.

Table 3 reflects delivery data obtained via chart review. Mean gestational age at delivery was 39.6 weeks. Mean duration of labor—defined as the time from first documentation of regular contractions plus cervical dilation to vaginal delivery—was 9 hours, with a range of 1 to 21 hours. Slightly more than half of women delivered vaginally, with the remaining having planned, emergency, or posttrial-of-labor (PTOL) cesarean sections. Infants had a mean gestational weight of 3406 grams, and most had five-minute Apgar scores of 10.

Forty-one percent of women had at least one birth complication. The most common complications were fetal distress (41%), preterm membrane rupture (26%), umbilical cord issues such as prolapsed, entanglement or nuchal cords (17%), and delayed labor (7%). 

With regard to Research Question 1, (*is optimism or pessimism associated with unplanned cesarean section delivery?*), bivariate analyses comparing optimism and pessimism against unplanned cesarean section indicated that both were significant: optimism (*P*  =  .047, 95% CI. 012, 1.81), pessimism (*P*  =  .003; 95% CI −2.42, −.529) (See Table 4). In addition, labor duration (*P*  =  .004, 95% CI 1. 009, 5.16) and the presence of birth complications (*P*  =  .01, Chi Square = 6.65) were also found to be significant. No other demographic or clinical factors were significantly associated with unplanned cesarean section. 

Table 5 Model 1, illustrates the findings with regard to Research Question 2 (*which is more strongly associated with unplanned cesarean section delivery, optimism or pessimism?*). In an unadjusted model in which both optimism and pessimism were regressed against unplanned cesarean section, pessimism remained statistically significant while optimism failed to meet the threshold for statistical significance. (pessimism OR = 1.28, 95% CI: 1.06, 1.56, *P*  =  .01; optimism OR = 0.88, 95% CI: 0.71, 1.08; *P*  =  .22).

When the same model was then adjusted for a variety of clinical factors (see Table 5 Model 2) to answer Research question 3 “*if there is a significant relationship between optimism, pessimism, and unplanned cesarean section delivery, is that relationship robust enough to remain significant when clinical factors are included in the model?”*, pessimism remained significantly associated with unplanned cesarean section (OR = 1.42; 95% CI: 1.11, 1.81; *P*  =  .004). Of note, labor duration and birth complications (preeclampsia, intrauterine infection, breech presentation, delayed labor, etc.) were the only clinical factors in the adjusted model that had a significant relationship to unplanned cesarean section delivery.

## 4. Discussion

This study showed an association between higher levels of generalized maternal pessimism during pregnancy and an increased likelihood of an unplanned c-section delivery among women presenting for prenatal care and delivering their infants at a tertiary care hospital in Beijing, China. This association was robust enough to remain, even when adjusted for clinical factors likely to be linked to a risk of unplanned cesarean section delivery. Interestingly, pessimism not optimism remained significant throughout the analysis. 

However, what is not clear, and what the cross-sectional study design of the study does not allow us to explore, is the mechanism of action. What is it about being pessimistic that is related to unplanned c-section delivery? It is possible that pessimists have qualitatively different or less effective coping skills than their less pessimistic counterparts [47–50]. Additionally pessimists, by virtue of believing that negative outcomes are likely, may be more fearful during labor. Emotional factors such as fear of delivery or fear of pain [51] have been linked to increased risk of c-section. Pessimists may also be more likely than their optimistic counterparts to abandon a traditional vaginal delivery and opt for a c-section if given the opportunity. Conceivably pessimism may serve as a proxy for another latent variable. Previous studies have linked optimism and pessimism to age, spirituality, and even SES, [52–54] but an additional, as yet undescribed and measured variable could explain the relationship between pessimism and unplanned cesarean section rates.

By contract, optimists have been found to be more likely to adopt active coping strategies and reappraise a situation in a positive way if an important goal is blocked [50]. It is possible that such coping strategies may allow optimists to relax during delivery more easily than their more pessimistic peers, reducing the likelihood of “failure to progress.” Our findings do not support this possibility: pessimism showed a significant association with unplanned cesarean section deliveries, while levels of optimism did not. This is not only useful in reaffirming that optimism and pessimism are two separate constructs rather than poles on a continuum [55, 56], but is also instructive in potential interventions during pregnancy. Encouraging positive thoughts may not be nearly as helpful as discouraging negative ones. 

The idea that cognitive predispositions that precede delivery may be associated with type of delivery is worthy of further exploration—including whether interventions can be designed to influence women's predispositions. For example, could cognitive behavioral therapy be used to reframe pessimists' negative thoughts, and might that result in lower cesarean-section rates? Perhaps more fundamentally, can pessimism be unlearned? 

Despite a dearth of information on pessimism, research suggests that optimism can be learned and practiced [57]. Avoiding negative environments, seeking the company of positive individuals and reframing challenges as opportunities are some of the ways experts suggest “activating” one's optimism [57]. Yet it is unclear whether such techniques would be effective enough to impact health outcomes.

Nevertheless, our findings are noteworthy for two reasons. First, they demonstrate the potential relationship/association between psychological factors assessed during pregnancy and eventual delivery outcomes, and second, they illustrate the potential strength of psychological factors such as pessimism.

That birth complications were significantly associated with unplanned cesarean sections is to be expected—given that complications such as fetal distress, preeclampsia, prolonged/obstructed labor, or shoulder dystocia are primary indications for cesarean section delivery [8, 24]. It is also not surprising that duration of labor is associated with unplanned cesarean section. We also observed that women who delivered vaginally in this sample had longer labors than those who had unplanned cesarean sections (data not shown). It was interesting to note that in this study the length of time women were allowed to attempt labor before a cesarean section was chosen was much shorter than in the United States (average unplanned cesarean section labor duration in this study was 3.5 hours, compared to 16.0 hours among nulliparas and 12.4 hours among multiparas in the United States [58]).

### 4.1. Limitations

There are several limitations to this study. First, the use of the LOT-R has not been formally validated among Chinese pregnant women. However, the instrument has been used repeatedly in China [39–46, 59] and it was carefully pretested in this population prior to study implementation. Our focus groups and pilot testing did not indicate any difficulties in interpretation of these items. Nonetheless, the instrument may benefit from a more rigorous validation study in this population. Also, the use of a cross-sectional convenience sample that includes mostly primiparous women limits inference to a wider population of pregnant Chinese women. In this study, all women presenting to the clinic were asked to participate, and it is possible that the women presenting during this study period were different from the larger population of pregnant women in Beijing. Future studies would benefit from a design that includes random selection at a variety of institutions across Beijing and across China.

This study also includes women in their last trimester of pregnancy. Although optimism/pessimism is considered a stable construct, it would be valuable to determine the potential impact of earlier recruitment.

This study also reveals what some would call excessively high episiotomy, cesarean section, and forceps rates, limiting its generalizability to settings without similar rates. Nonetheless, we believe these findings reflect clinical practice at one large tertiary care center in China, and as such provide valuable insight. 

Finally, this study asked women to self-report their pregnancy complications. It was not possible to verify these self-reports against medical records data. We were able to elicit birth complications from the medical record, but this study relies upon self-reported complications during the gestation period. We do not believe this to be a significant limitation, however, given the high probability that women will know whether they are experiencing nausea, vomiting, or abdominal pain, or whether they have vaginal bleeding or swollen hands and feet. We also expect that women will remember if a doctor has told them they have high blood pressure, gestational diabetes, or other more serious pregnancy complications.

### 4.2. Conclusions and Potential Implications

This research has several important implications. First, it confirms what many women and practitioners may have believed anecdotally: that a woman's mindset during her pregnancy may have an impact on her delivery. It also raises questions about the value of positive thinking—the predominant advice given to pregnant women—versus the value of not thinking negatively. Second, it raises important questions about whether inexpensive cognitive behavioral therapy or other mindset-altering interventions among pregnant women could be used to reduce unplanned cesarean section rates.

More research is needed to elucidate the relationship between pessimism and pregnancy outcomes. Is this study replicable? Is the finding real, or is it masking some other yet to be determined variable? Is a negative outlook merely associated with a risk of unplanned cesarean section delivery, or can a causal pathway be identified? In addition, is it possible to change women's levels of pessimism? And would interventions to decrease pessimism translate to reduced rates of c-sections? 

These are just some of the questions in need of answers as researchers continue to explore the relationship between psychosocial variables and pregnancy outcomes.

**Current Knowledge on This Subject**

- Cesarean section rates are rising, due, in large part, to nonclinical factors.
- Physician factors, insurance status, hospital policies, and maternal preferences are all non-clinical factors that influence csection rates.
- Maternal cognitive predispositions during pregnancy (specifically optimism/pessimism) have not been examined in relationship to unplanned cesarean section deliveries.

**What This Study Adds**

- Pessimism during pregnancy appears to be associated with an increased risk of unplanned cesarean section delivery in this population.
- Pessimism during pregnancy remains associated even when clinical factors are controlled.
- Pessimism appears to be a stronger correlate than optimism—suggesting that having positive thoughts/expectations may not be as helpful as not having negative thoughts/expectations during pregnancy.

## Figures and Tables

**Table 1:** Demographic characteristics of study participants versus those excluded due to incomplete data.

Variable	Included women (*N* = 141)	Excluded women* (Total *N* = 86)	*P*-value
	mean (± SD)	mean (± SD)	
Age	30.0 years (±3.3)	29.8 years (±3.5)	*P* = .682 (NS)
		Missing = 5	

Weeks pregnant at enrollment	35.6 (±2.5)	35.3 (±2.5)	*P* = .345 (NS)
		Missing = 2	

	*N* (Percent)	*N* (Percent)	

Ethnicity	Han 128 (93.4)	Han 78 (91.8)	*P* = .695 (NS)
	Hui 2 (1.5)	Hui 2 (2.4)	
	Xian 1 (0.7)	Xian 0 (0)	
	Man 3 (2.2)	Man 1 (1.2)	
	Other 3 (2.2)	Other 4 (4.7)	
	Missing = 4	Missing = 1	

Highest level of education	HS grad or less 19 (13.5) College Grad or less 90 (63.8) Graduate/Professional Degree or less 32 (22.6)	HS grad or less 23 (27.3) College Grad or less 51 (60.7) Graduate/Professional Degree or less 10 (11.9)	*P* = .012*
		Missing = 2	

Family income per month (Chinese Yuan)	3000 or less 19 (13.4)	3000 or less 19 (22.4)	*P* = .106 (NS)
	3001–5000 36 (25.7)	3001–5000 25 (29.4)	
	5001–10000 56 (40.0)	5001–10000 31 (36.5)	
	>10001 30 (21.4)	>10001 10 (11.8)	
		Missing = 1	

Married		84 (98.8)	*P* = .197 (NS)
	141 (100.0)	Missing = 1	

Originally from Beijing		38 (44.7)	*P* = .997 (NS)
	63 (44.7)	Missing = 1	

Owns a car		38 (45.7)	*P* = .638 (NS)
	60 (42.5)	Missing = 3	

Worked for money before delivery	131 (92.9)	73 (87.9)	*P* = .209 (NS)
		Missing = 3	

Intends to work for pay after delivery	134 (95.0)	76 (91.5)	*P* = .300 (NS)
		Missing = 3	

* Women with incomplete baseline data were excluded from the regression analysis. Key variables for inclusion were age, education, income, number of previous deliveries, originally from Beijing (y/n), car ownership (y/n), work before pregnancy (y/n), intend to work after pregnancy (y/n), insurance status, previous abortion (y/n), previous miscarriage (y/n), and experience of this pregnancy.

**Table 2:** Self-reported health-related variables collected during pregnancy from participants versus those excluded due to incomplete data.

Variable	Included women (*N* = 141)	Excluded women* (Total *N* = 86)	*P*-value
	*N* (Percent)	*N* (Percent)	
One or more previous pregnancies	82 (58.5)	46 (55.4)	*P* = .463 (NS)
	Missing = 1	Missing = 3	

One or more previous deliveries	7 (5.0)	8 (9.8)	*P* = .168 (NS)
		Missing = 4	

Previous abortion		42 (57.5)	*P* = .774 (NS)
	84 (59.5)	Missing = 13	

Number of abortions	0 : 41 (33.1)	0 : 26 (37.7)	*P* = .416 (NS)
	1 : 57 (46.0)	1 : 26 (37.7)	
	2 : 22 (17.7)	2 : 11 (15.9)	
	3+ : 4 (3.2)	3+ : 6 (8.9)	
	Missing = 17	Missing = 17	

Previous miscarriage		8 (12.1)	*P* = .161 (NS)
	9 (6.3)	Missing = 20	

Trouble getting pregnant (> 12 mo to conceive)	34 (24.3)	29 (35.4)	*P* = .077 (NS)
	Missing = 1	Missing = 4	

Used fertility treatment	7 (5.0)	9 (10.7)	*P* = .108 (NS)
	Missing = 1	Missing = 2	

Experience with current pregnancy	No complications 101 (71.6)	No complications 40 (69.0)	*P* = .116 (NS)
	Somewhat easy 36 (25.5)	Somewhat easy 12 (20.7)	
	Somewhat difficult 4 (2.8)	Somewhat difficult 5 (8.6)	
	Extremely difficult 0 (0)	Extremely difficult 1 (1.7)	

Medical insurance	Gov't issued 85 (60.2)	Gov't issued 40 (50.0)	*P* = .316 (NS)
	Employer or private	Employer or private	
	Insurance 46 (32.5)	Insurance 29 (46.3)	
	No insurance 10 (7.1)	No insurance 11 (13.7)	
		Missing = 6	

Seen a doctor, counselor, or other professional for emotional issues	Ever 5 (3.5)	4 (4.8)	*P* = .653 (NS)
	Currently 0 (0)	3 (3.6)	*P* = .024*

Presence of nonpregnancy-related health problems		3 (3.7)	*P* = .960 (NS)
	5 (3.5)	Missing = 5	

*P < 0.05

**Table 3:** Postdelivery data retrieved from the medical record regarding pregnancy and delivery (*N* = 141).

Variable	Mean (± SD)
Number of weeks pregnant at delivery	39.6 (± 1.2)

Labor duration (vaginal deliveries only)	8.96 hrs (± 4.3)
	Range: 1.0–20.8 hours

Mean birthweight (grams)	3406.2 (± 416.3)

	*N* (Percent)

Percent w/live Birth	141 (100)

Percent w/Apgar <10	1 minute: 6 (4.3)
	5 minute: 1 (0.7)
	Missing = 1

Birth types	Vaginal 81/141 (57.4)
	Episiotomy 61/81 (75. 3)
	Forceps 16/81 (19.7)
	Cesarean 67/141 (47.5)
	Planned 41/67 (61.2)
	Emergency 25/67 (37.3)
	After TOL 11/67 (16.4)
	Both 7/141 (5.0)

Most common pregnancy complications	Anemia 26 (18.4)
	Gestational diabetes 13 (9.2)
	Elderly primigravida 9 (6.4)
	IntraUterine Infection 8 (5.7)
	Macrosomia 8 (5.7)


Most common delivery/birth complications	Fetal Distress 58 (41.1)
	Preterm Mem. rupture 36 (25.5)
	Umbilical cord 24 (17.0)
	Delayed labor 10 (7.1)
	Hemorrhage 5 (3.5)
	Preeclampsia 5 (3.5)
	Preterm labor 2 (1.4)

Number of delivery complications	0 complications: 45 (31.9)
	1 of the above: 61 (43.3)
	2 of the above: 29 (20.6)
	3+ of the above: 6 (4.3)

**Table 4:** Bivariate comparisons of key variables against unplanned c-section (*N* = 141).

Predictor	Statistic	*P*-Value (95% CI)
Number of pregnancy complications	*t* = −.010	0.992 (−.41,.41)

Number of pregnancy complications that are linked to risk of C-Section	*t* = 0.353	0.725 (−.20,.29)

Number of pregnancy complications that are not linked to risk of C-section	*t* = −.292	0.771 (−.36,.27)

Labor duration	*t* = 2.93	.004* (1.009, 5.16)

Infant birthweight	*t* = −1.58	0.116 (−315.47, 34.9)

Gestational age	*t* = −.269	0.789 (−.57,.43)

Maternal age	*t* = .612	0.541 (−.97, 1.85)

Optimism subscale	*t* = 2.004	0.047* (.012, 1.81)

Pessimism subscale	*t* = −3.077	0.003* (−2.43 −.529)

Previous abortion	Chi Square = .159	0.690

Previous miscarriage	Chi Square = .059	0.809

Nonpregnancy-related health issues	Chi Square = 1.42	0.232

Perception of pregnancy experience	Chi Square = .098	0.952

Birth complications	Chi Square = 6.65	0.010*

Education	Chi Square = .307	0.858

Income	Chi Square = 3.638	0.303

Insurance	Chi Square = 5.229	0.073

*P < .05.

**Table 5:** Logistic regression analyses exploring predictors of unplanned cesarean section in China^1^.

	Model 11			Model 22		
	AUC = 0.70			AUC = 0.86		
	Odds Ratio (Exp(B))	95% CI	*P*-Value	Odds ratio (Exp(B))	95% CI	*P*-Value
Pessimism	1.28	1.06, 1.56	.01*	1.45	1.11,1.81	.001*

Optimism	.880	0.72, 1.08	.22 (NS)	.847	0.66, 1.09	.20 (NS)

Birth complications	—	—	—	15.36	3.07, 76.96	.001*

Labor duration	—	—	—	.809	0.71, 0.92	.001*

^1^Unadjusted pessimism and optimism regressed against unplanned cesarean section delivery (yes/no).

^2^Optimism and pessimism adjusted for previous abortion, previous miscarriage, pregnancy complications, infant gestational age at delivery, infant birthweight, labor duration, birth complications, and self-rated difficulty of this pregnancy. Birth complications and labor duration were the clinical factors that were significantly associated with unplanned cesarean section delivery (*P* =  .001).

*P ≤ .01.
